The article "miR-641 Inhibited Cell Proliferation and Induced Apoptosis by Targeting NUCKS1/PI3K/AKT Signaling Pathway in Breast Cancer" was published in 2022. Journal: Comput Math Methods Med.

# miR-641 Inhibited Cell Proliferation and Induced Apoptosis by Targeting NUCKS1/PI3K/AKT Signaling Pathway in Breast Cancer

**DOI:** 10.1155/2022/5203839

**Published:** 2022-01-12

**Authors:** Li Li, Da Wei, Junying Zhang, Rong Deng, Jinhai Tang, Dongming Su

**Affiliations:** ^1^Department of General Surgery, Nanjing Medical University Affiliated Cancer Hospital Cancer Institute of Jiangsu Province, Baiziting 42, Nanjing 210009, China; ^2^The Fourth Clinical School of Nanjing Medical University, Nanjing 210009, China; ^3^Center of Clinical Laboratory, Cancer Institute of Jiangsu Province, Nanjing Medical University Affiliated Cancer Hospital, Nanjing, China; ^4^Department of General Surgery, The First Affiliated Hospital with Nanjing Medical University, Nanjing, Jiangsu, China; ^5^Center of Metabolic Research, Nanjing Medical University, Nanjing, China

## Abstract

**Objective:**

Studies revealed an important role of microRNAs (miRNAs) in multiple cancers, including breast cancer. In the present study, we evaluated the role and function of miR-641 in breast cancer.

**Methods:**

The expression level of miR-641 in breast cancer cell lines (Hs-578T, MCF7, HCC1937, and MAD-MB-231) was determined by real-time PCR. Functional analyses, including CCK-8 assay, transwell assay, wound-healing assay, and apoptosis detection, were carried out to explore the roles of miRNA-641 in malignant behaviors of breast cancer. Luciferase report assay was used to investigate the regulatory association of miRNA-641 with its potential targets.

**Results:**

The expression levels of miR-641 were downregulated, while the expression levels of nuclear casein kinase and cyclin-dependent kinase substrate 1 (NUCKS1) were increased in breast cancer cell lines. The *in vitro* results showed that miR-641 repressed proliferation and migration/invasion and promoted apoptosis of breast cancer cells. NUCKS1, a positive regulator of phosphatidylinositol-3-kinases (PI3K)/protein-serine-threonine kinase (AKT) pathway, was confirmed as a direct target of miR-641. The of treatment of the PI3K agonist, 740Y-P, could abrogate the antioncogenic potentials of miR-641 in breast cancer cells.

**Conclusion:**

miR-641 functioned as a tumor suppressor through the PI3K/AKT signaling pathway via targeting NUCKS1 in breast cancer.

## 1. Introduction

Breast cancer is one of the widely occurred inducers of cancer worldwide and the second primary cause of cancer mortality amid women. Mortality exhibited a main association with the development of metastases. The incidence of breast cancer in women is getting higher and higher, constituting a major public health problem. Even if the prognosis is excellent when the cancer is located in the breast (5-year survival rate, 99%), in the case of disseminated disease, the survival rate will drop rapidly (if there is distant metastasis, the survival rate is 26%). Breast cancer can be classified into noninfiltrating carcinoma, invasive lobular carcinoma, metaplastic carcinoma, tubular carcinoma, invasive ductal carcinoma, and mucinous carcinoma according to the latest 5^th^ edition of the World Health Organization (WHO) histopathologic classification [1]. The surgical resection is the primary curative treatment for early-stage breast cancer [2]. Hormone treatments and CDK 4/6 inhibitors are widely employed in metastatic hormone receptor-positive setting, following the outstanding results of phase III clinical trials [3]. More recently, immunotherapy has emerged as a valuable treatment option in triple-negative breast cancer [4]. The cumulative results showed that the T lymphocyte infiltration of triple-negative breast cancer (TNBC) and human epidermal growth factor receptor 2 (HER2) breast cancer was higher than that of estrogen receptor-positive and HER2 negative breast cancer. Immunotherapy has shown good results in TNBC, but in order to improve the clinical benefit of immunotherapy for breast cancer, it is necessary to develop immunooncology combination therapy [5–7]. Although the use of adjuvant chemotherapy and hormone drugs has increased the mortality rate of breast cancer, it is still challenging to determine who will benefit from these treatments and who may be exposed to toxicity [8–11]. With the rising cost of health care and the introduction of new targeted therapies, biomarkers have been used as a means of assisting breast cancer diagnosis, prognosis, response prediction, and disease surveillance during and after treatment. Prognostic and therapeutic biomarkers, their utility in breast cancer management, and current recommendations on their clinical use should be paid attention [12–14].

The article "miR-641 Inhibited Cell Proliferation and Induced Apoptosis by Targeting NUCKS1/PI3K/AKT Signaling Pathway in Breast Cancer" was published in 2022. Journal: Comput Math Methods Med.

MicroRNAs (miRNAs) are small noncoding RNA molecules of about 18 to 25 nucleotides in length that inhibit gene expression at the posttranscriptional levels [15–18]. miRNAs bind to their target mRNAs, leading to the degradation or the translational suppression of target mRNAs [19]. miRNAs affect many important biological activities and control cell growth, differentiation, proliferation, and apoptosis [20]. In human cancers, the expression of abnormal miRNAs is more frequent and plays an important role in the occurrence and development of cancer. Kong et al. [19] demonstrated that miRNA-140-3p inhibits the proliferation, migration, and invasion of lung cancer cells by targeting ATP6AP2. Therefore, it is necessary to evaluate the influence of the abnormal expression of miRNA in cancer. The tumor suppressor effect of miR-641 has been proposed in a previous study: Yao et al. [20] showed that the overexpression of miR-641 inhibited the proliferation of cervical cancer cells. According to the research of Richards et al. [21], inhibiting miR-641 makes tumor cells sensitive to cisplatin-induced apoptosis. miRNA-641 is located at chromosome 13q14 that functions as a tumor suppressor in different types of cancers including lung cancer [22], cervical cancer [23], and osteosarcoma [24]. However, the role of miR-641 in breast cancer has not been studied. As far as we know, this is the first study to evaluate the roles of miR-641 in breast cancer.

## 2. Materials and Methods

### 2.1. Cell Culture

Human Hs-578T, MCF7, HCC1937, and MAD-MB-231 breast cancer cells and human breast epithelial MCF-10A cells were obtained from American Type Culture Collection (ATCC, Rockville, MD, USA). MCF-10A cells were cultured in DMEM/F12 (1 : 1) medium (Gibco, USA), and MAD-MB-231 cells were cultured in Leibovitz's L-15 medium (Gibco, USA). The other cells were cultivated in DMEM containing 10% fetal bovine serum. The MycAway™ Plus-Color One-Step Mycoplasma Detection Kit was used to test the mycoplasma, and no mycoplasma contamination was found in the cells.

### 2.2. Cell Transfection and Treatment

MAD-MB-231 and MCF7 cells in the logarithmic growth phase were transfected with either miR-641 mimics or mimic negative control (mimic NC) (GenePharma), following 1.5 h of treatment with 50 *μ*g/ml 740Y-P (Sigma-Aldrich, St. Louis, MO, USA), a PI3K agonist. Transfection efficiency was assessed by real-time PCR and qualitative analyses of green fluorescent protein (GFP).

### 2.3. Bioinformatics Analysis

The target gene of miR-641 was predicted using TargetScan and miRanda softwares. Whether NUCKS-1 was the target gene of miR-641 was measured by TargetScan software. In addition, whether NUCKS-1 could combine with miR-641 was analyzed by miRanda software [25].

### 2.4. Luciferase Reporter Assay

WT- and MUT-NUCKS1-3′UTR luciferase reporter plasmids were obtained from Promega (Madison, WI, USA). The cells were inoculated into a 12-well plate. When the cell confluence was approximately 70%, the WT- or MUT-NUCKS1-3′UTR was transfected into the cells. After 24 hours, luciferase signals were measured with Dual-luciferase Reporter Assay System using a TECAN Infinite F500 platform.

### 2.5. RNA Pull-Down

RNA pull-down was conducted in MAD-MB-231 and MCF7 cells (1 × 10^4^) using the Magnetic RNA-Protein Pull-Down Kit (Pierce Biotechnology, Rockford, IL, USA) in accordance with the manufacturer's instructions. miR-641 probe and NC probe are constructed by sigma. The cells were harvested and lysed, and the supernatant was obtained by centrifugation (5000 rpm/min, 10 min). miR-641 probe and NC probe were incubated with a supernatant at 37°C overnight. The magnetic beads (Pierce Biotechnology) were then added to the supernatant and incubated for 1 h at 37°C to allow the beads to adsorb the probe. After cleaning, the mRNA binding to the probe was harvested. The relative NUCKS1 expression was analyzed by real-time PCR assay.

The article "miR-641 Inhibited Cell Proliferation and Induced Apoptosis by Targeting NUCKS1/PI3K/AKT Signaling Pathway in Breast Cancer" was published in 2022. Journal: Comput Math Methods Med.

### 2.6. Real-Time PCR

Total RNA from cells was isolated by Trizol Reagent (Life Technology) and was reversely transcribed into cDNA using the TaqMan microRNA Reverse Transcription Kit (Life Technology). The amplification of miR-641 was performed with the TaqMan Universal PCR Master Mix II (Life Technology) using the 7500 FAST real-time PCR System (Applied Biosystems, Carlsbad, CA, USA), with U6 as an endogenous control. The PCR primers used in this case were as follows: miR-641 forward, 5′-TTATACTCTCACCATTTGGATC-3′, reverse, 5′-TGACAAGATTTTACATCAAGAA-3′; U6 forward, 5′-CTTCGGCAGCACATATACT-3′, reverse, 5′-AAAATATGGAACGCTTCACG-3′. The forward and reverse primers for NUCKS1 were 5′-GGCCTGTCAGAAATAGGAAGGT-3′ and 5′-TTTAGCTTCTCGGGGAGATGAT-3′. GAPDH was used as the endogenous control. The primers for GAPDH were 5′-CGGAGTCAACGGATTTGGTCGTAT-3′ (forward) and 5′-AGCCTTCTCCATGGTGGTGAAGAC-3′ (reverse).

### 2.7. Western Blot

Immunoblotting was conducted in cultured cells according to the standard procedures as previously described [26]. Total proteins were obtained from cells with RIPA Reagent (Sigma). Equal amounts of protein (20 *μ*g) were separated with 12% SDS-PAGE, then transferred to PVDF membranes (Millipore). After that, the membranes were incubated in 5% nonfat milk for 1 h at room temperature and then treated with the primary antibodies overnight at 4°C. After being washed for 3 times, the membranes were incubated with second antibody (1 : 5000, ab150077 or ab150113, Abcam) for 1 h at room temperature. Finally, the protein bands were detected using an ECL detection system (Thermo). The data were analyzed using ImageJ software (NIH).

The antibodies used in this analysis included rabbit polyclonal to NUCKS1 (ab7770), proliferating cell nuclear antigen (PCNA; ab15212), Ki67 (ab15580), Bax (ab53154), Bcl-2 (ab196495), caspase-3 (ab13847), caspase-9 (ab52298), Cyclooxygenase-2 (Cox-2; ab15191), matrix metallopeptidase-2 (MMP-2; ab97779), MMP-9 (ab38898), phosphatidylinositol-3-kinases (PI3K; ab70912), p-PI3K (ab138364), protein-serine-threonine kinase (AKT; ab8805), and p-AKT (ab38449), purchased from Abcam (Cambridge, UK). GAPDH was used as a loading control.

The article "miR-641 Inhibited Cell Proliferation and Induced Apoptosis by Targeting NUCKS1/PI3K/AKT Signaling Pathway in Breast Cancer" was published in 2022. Journal: Comput Math Methods Med.

### 2.8. Immunofluorescence

After being fixed with 4% paraformaldehyde for 10 min and permeabilized by 0.3% Triton X-100 for 15 min, MAD-MB-231 and MCF7 cells cultured on glass coverslips were incubated with 3% BSA for 30 min at room temperature to block nonspecific binding. Following that, cells were stained with p-PI3K and p-AKT antibodies overnight at 4°C and fluorescein isothiocyanate- (FITC-) labeled secondary antibodies (1 : 500, ab7086, Abcam) for 2 h at room temperature. Then, the nucleus was counterstained with Hoechst 33258 (Sigma, USA) for 30 min. Cells were photographed under a fluorescent microscope (Leica, Germany).

### 2.9. Proliferation Assay

For CCK-8 assay, cells were seeded into 96-well plates at a density of 2 × 10^3^ cells/well, and then, CCK-8 reagent (Beyotime, Shanghai, China) was added at 0 h, 24 h, 48 h, and 72 h. Absorbance was detected at 450 nm after incubation for another 2 h. For EdU assay, transfected cells were incubated with EdU solution for 2 h, fixed for 30 min with 4% paraformaldehyde, and stained with KFluor488 EdU kit (Life Technologies) according to the manufacturer's instructions. For colony formation assay, transfected cells were reseeded onto 6-well plates, fixed with 4% paraformaldehyde for 15 min, and subsequently stained with 0.1% crystal violet. The number of colonies was analyzed using an optical microscope.

### 2.10. Apoptosis Detection

Apoptosis was assessed using the Annexin V-FITC Apoptosis Detection Kit (Biosea, Beijing, China). After transfection, MAD-MB-231 and MCF7 cells (1 × 10^4^) were fixed with ethyl alcohol at 4°C for 2 h. After the addition of propidium iodide (PI) and FITC Annexin V at 4°C under darkness for 30 min, the apoptotic cells were detected by flow cytometry.

### 2.11. Wound-Healing Assay

Cell migration capacity was measured by wound-healing assay. Transfected cells were seeded in 6-well plates. After cellular fusion, the cell monolayer was scraped using a sterile 200 *μ*l pipette tip to create separate wounds, and the medium of serum-free was used to incubate the wounds at 37°C for 48 h. The results were photographed under a microscope (Olympus, Tokyo, Japan) at 0 h and 48 h after wounding.

### 2.12. Transwell Assay

Cell invasion capacity was measured with a transwell chamber (Millipore). For the invasion assay, the upper chamber of every insert was coated with Matrigel (BD biosciences). Cells (5 × 10^4^/ml) cultured with serum-free medium were added into the upper chamber, and medium with 20% FBS was added into the lower chamber. For the migration assay, cells (5 × 10^4^/ml) were added into the upper chamber inserts with serum-free medium. The lower chambers contained medium with 20% FBS. After 24 h incubation, cells at the bottom of the membrane were fixed with 4% polyoxymethylene for 15 min and then stained with 0.1% crystal violet dye for 10 min at 37°C. The results were visualized under a light microscope (×400 magnification) in 5 randomly selected fields of view after being stained with 4% crystal violet.

The article "miR-641 Inhibited Cell Proliferation and Induced Apoptosis by Targeting NUCKS1/PI3K/AKT Signaling Pathway in Breast Cancer" was published in 2022. Journal: Comput Math Methods Med.

### 2.13. Statistical Analysis

One-way ANOVA (analysis of variance) was used to analyze difference among groups using GraphPad prism version 7.0 (GraphPad Software, San Diego, CA, USA), and post hoc test (Tukey) was performed after ANOVA. All results were expressed as mean ± standard deviation (SD), and values of *P* < 0.05 were considered statistically significant. In our experiment, the sample size of each group was set to *n* = 5.

## 3. Results

### 3.1. The Expression Levels of miR-641 Are Decreased in Breast Cancer Cells

By using real-time PCR assay, we assessed the miR-641 expression in 4 human breast cancer cell lines (Hs-578T, MCF7, HCC1937, and MAD-MB-231). Compared with MCF-10A cells, miR-641 expression was significantly downregulated (Figure 1(a)). Given that the expression levels of miR-641 in MDA-MB-231 and MCF7 cells were lower expressed than those in Hs-578T and HCC1937, MDA-MB-231 and MCF7 cells were used for the following experiments.

### 3.2. miR-641 Inhibits the Proliferation of Breast Cancer Cells and Promotes Apoptosis

To investigate the functional roles of miR-641 in breast cancer cells, we used the miR-641 mimic to overexpress the miR-641 in MDA-MB-231 and MCF7 cells. Transfection efficiency was confirmed by RT-PCR and fluorescence quantification of GFP. We showed that miR-641 mimic transfection significantly increased the RNA levels of miR-641 and yielded GFP expression in MDA-MB-231 and MCF7 cells (Figures 1(b)–1(c)). CCK-8 assay elucidated that miR-641 mimic could significantly repress the viabilities of MDA-MB-231 and MCF7 cells in a time-dependent manner (Figure 1(d)). EdU incorporation assay revealed that miR-641 overexpression descended the numbers of EdU-positive cells (Figure 1(e)). The results of colony formation assay illustrated that the number of colonies was declined in response to the upregulation of miR-641 expression (Figure 1(f)). The influence of miR-641 expression on proliferation-associated genes (PCNA and Ki67) was further analyzed by western blotting. As indicated in Figure 1(g), forced expression of miR-641 observably downregulated the protein levels of PCNA and Ki67 in MDA-MB-231 and MCF7 cells. Flow cytometry analyses revealed that the percentage of apoptotic cells was increased by overexpression of miR-641 (Figure 2(a)). Consistently, the expression levels of proapoptotic proteins (Bax, caspase-3, and caspase-9) were all correspondingly increased, whereas Bcl-2, the antiapoptotic gene, was markedly downregulated in miR-641-overexpressed MDA-MB-231 and MCF7 cells (Figure 2(b)).

The article "miR-641 Inhibited Cell Proliferation and Induced Apoptosis by Targeting NUCKS1/PI3K/AKT Signaling Pathway in Breast Cancer" was published in 2022. Journal: Comput Math Methods Med.

### 3.3. miR-641 Suppresses the Migration and Invasion of Breast Cancer Cells

Furthermore, ectopic expression of miR-641 limited the migratory and invasion capabilities of MDA-MB-231 and MCF7 cells (Figures 3(a) and 3(b)). We found that the overexpression of miR-641 expression led to significant decreases in the protein expression levels of Cox-2, MMP-2, and MMP9, which were the crucial indicators of cancer metastasis (Figure 3(c)).

### 3.4. NUCKS1 Is a Direct Target of miR-641 in Breast Cancer Cells

As is known to all, miRNAs have multiple biological functions through targeting various mRNAs. To elucidate the underlying antitumor mechanisms of miR-641 in human breast cancer cells, we used bioinformatics programs to identify potential target genes of miR-641. NUCKS-1 was predicted to be the target gene of miR-641 in TargetScan software. In addition, through the analysis of NUCKS-1 in miRanda software, we found that miR-641 had the same binding site with NUCKS-1 (Figure 4(a)). The luciferase reporter assay showed that overexpression of miR-641 repressed the relative luciferase activities containing the wild-type 3′-UTR of NUCKS1 but had no obvious effect on mut 3′-UTR of NUCKS1 (Figure 4(b)). Accordingly, miR-641 was found to physically interact with NUCKS1 as demonstrated by biotinylated-miRNA pull-down using biotin-labeled miR-641 (Figure 4(c)). In addition, ectopic expression of miR-641 suppressed the mRNA and protein expression of NUCKS1 in MDA-MB-231 and MCF7 cells (Figures 4(d) and 4(e)). By using real-time PCR and western blotting assays, we assessed the NUCKS1 expression in breast cancer cell lines (Hs-578T, MCF7, HCC1937, and MAD-MB-231). Compared with MCF-10A cells, NUCKS1 mRNA and protein expression was significantly upregulated (Figures 4(f) and 4(g)).

### 3.5. Overexpression of miR-641 Inactivates the PI3K/AKT Signaling Pathway

NUCKS1 is a critical regulator of PI3K/AKT signaling, which prompts us to determine whether dysregulation of miR-641 could alter the activity of PI3K/AKT signaling in breast cancer cells. The western blotting results showed that overexpression of miR-641 significantly decreased the protein phosphorylation levels of PI3K and AKT, but not their total protein expression in MDA-MB-231 and MCF7 cells (Figure 5(a)). As demonstrated by immunofluorescence staining, the PI3K and AKT phosphorylation in breast cancer cells was inhibited by miR-641 overexpression (Figure 5(b)).

The article "miR-641 Inhibited Cell Proliferation and Induced Apoptosis by Targeting NUCKS1/PI3K/AKT Signaling Pathway in Breast Cancer" was published in 2022. Journal: Comput Math Methods Med.

### 3.6. PI3K/AKT Signaling Pathway Mediates the Effect of miR-641 on the Breast Cancer Cells

Next, we examined whether the activation of PI3K/AKT signaling was critical for miR-641-mediated anticancer function. Transfected cells were exposed to PI3K activator (740Y-P) to verify the regulatory pathway. As shown in Figures 6(a)–6(c), 740Y-P treatment abolished miR-641 overexpression-induced proliferation inhibition of MCF7 cells. Moreover, 740Y-P attenuated MCF7 cell apoptosis induced by miR-641 overexpression (Figure 6(d)). Additionally, compared with the miR-641 mimic-treated group, 740Y-P treatment increased cell migration and invasion of MCF7 cells (Figures 6(e) and 6(f)). Thus, miR-641 exerted its function in breast cancer cells by inhibition of the PI3K/AKT signaling pathway. The expression levels of PI3K/AKT-related proteins were assessed using western blot (Figure 6(g)).

### 3.7. NUCKS1 Overexpression Antagonizes the Effect of miR-641 on the PI3K/AKT Signaling Pathway of Breast Cancer Cells

To further identify the mediatory role of NUCKS1 in linking the effect of miR-641 on the breast cancer progression, we overexpressed the NUCKS1 in both MDA-MB-231 and MCF7 cells. The overexpression efficiency is presented in Figure 7(a). We found that NUCKS1 overexpression significantly retarded the inhibitory effects of miR-641 mimic on the proliferation of MDA-MB-231 and MCF7 cells as evidenced by CCK-8 and EdU assays (Figures 7(b) and 7(c)). In contrast, forced expression of NUCKS1 decreased the miR-641 mimic-induced apoptosis of MDA-MB-231 and MCF7 cells (Figure 7(d)). Consistently, transwell assay revealed that NUCKS1 overexpression partially blocked the antimigration and anti-invasion effects of miR-641 on the breast cancer *in vitro* (Figure 7(e)). The western blotting results indicated that overexpression of miR-641 significantly decreased the protein phosphorylation levels of PI3K and AKT, but not their total protein expression in MDA-MB-231 and MCF7 cells, while NUCKS1 obviously restored the inhibitory effects of miR-641 mimic on the expression levels of PI3K/AKT-related proteins (Figure 8).

## 4. Discussion

In the present research, we confirmed that miR-641 expression was downregulated in breast cancer cells. Additionally, overexpression of miR-641 markedly reduced cell viability, migration, and invasion, while it promoted apoptosis. Furthermore, miR-641 was shown to be involved in the modulation of PI3K/AKT signaling by directly targeting NUCKS1. Abnormal expression of miRNAs could act as crucial biomarkers for diagnosis, therapy, and prognosis of breast cancer [27]. The anticarcinogenic effects of miR-641 have been reported in solid tumors. For example, overexpression of miR-641 led to antiproliferation and proapoptosis effects in lung cancer cells [22]. Yao et al. uncovered that miR-641 functioned as a tumor suppressor in cervical cancer via downregulating transcriptional repressor ZEB1 [23]. Silencing of miR-641 promoted osteosarcoma cell proliferation and metastasis by targeting homeobox protein Hox-A9 (HOXA9) [24]. Yan *et al*. reported that cytochrome P-450 monooxygenase 3A4 (CYP3A4) could be directly regulated by miR-641 in human hepatoma HepaRG cells [28]. Chen *et al*. indicated that miR-641 significantly downregulated neurofibromin 1 (NF1), which contributed to erlotinib resistance in non-small-cell lung cancer cells [29]. In the present study, miR-641 was substantially downregulated in breast cancer cells, suggesting that miR-641 might be a tumor suppressor during the progression of breast cancer. Given that miR-641 was decreased in breast cancer cells, we hypothesized that miR-641 might suppress the malignant phenotypes of breast cancer cells. The results confirmed that overexpression of miR-641 markedly inhibited tumor cell viability and metastasis and enhanced apoptosis.

The article "miR-641 Inhibited Cell Proliferation and Induced Apoptosis by Targeting NUCKS1/PI3K/AKT Signaling Pathway in Breast Cancer" was published in 2022. Journal: Comput Math Methods Med.

NUCKS1 is ubiquitously expressed in all mammalian tissues and has been confirmed to be overexpressed in many cancers, especially malignant neoplasms [30]. NUCKS1 is a substrate for casein kinase 2 (CK2), cyclin dependent kinase-1 (Cdk1) and DNA-activated kinase in vitro and in vivo [30, 31]. NUCKS1 contribute to the susceptibility, occurrence, and development of several cancers and other diseases, suggesting that NUCKS1 could be a potent marker for such diseases. In skin tumors, high expression of NUCKS1 in the nuclei of squamous cell carcinoma (SCC) and basal cell carcinoma (BCC) cells is more common than Ki67 expression. NUCKS1 expression has been found to be much lower in benign keratoacanthoma (KA) than in malignant tumors [32]. In breast carcinoma, NUCKS1 exhibited higher expression than other investigated markers (including Ki67, estrogen receptor, progesterone receptor, human epidermal growth factor receptor 2, and cytokeratin 5/6) [33]. Additionally, NUCKS1 is also highly expressed in breast cancer with obesity [34]. As previously described, NUCKS1 could increase the invasiveness of gastric cancer cells through the PI3K/Akt/mTOR signaling pathway, and these effects are mediated by IGF-1R [35]. We also found that NUCKS1 was significantly upregulated in breast cancer cells, indicating that NUCKS1 might be an oncogene for breast cancer pathogenesis. The upregulation of miR-641 inhibited NUCKS1 expression at both mRNA and protein levels in breast cancer cells.

PI3K/AKT is a common signaling cascade that emerges as an important player in the pathogenesis of various tumors, including breast cancer [36]. Huang et al. previously reported that NUCKS1-mediated gastric cancer aggressiveness was associated with the activation of the PI3K/AKT/mTOR signaling pathway [35]. Of note, overexpression of miR-641 blocked the activation of the PI3K/AKT pathway. Further mechanistic analysis validated that treatment with the PI3K agonist, 740Y-P, abrogated the antitumor effects of miR-641 in breast cancer.

The article "miR-641 Inhibited Cell Proliferation and Induced Apoptosis by Targeting NUCKS1/PI3K/AKT Signaling Pathway in Breast Cancer" was published in 2022. Journal: Comput Math Methods Med.

However, some limitations still existed in this study. It is a limitation of this study that the relevant data of clinical samples are not used. Further experiments are needed to confirm the function of miR-641 *in vivo*. The underlying mechanism of the inhibition still remains to be investigated. Moreover, the lack of miR-641 inhibitor experiments on the cell lines with higher miR-641 expression levels (Hs-578T and HCC1937 cells) is a limitation in this paper, and we will explore that in the future. Besides, except for NUCKS upstream of PI3K, further experiments are needed to confirm whether miR-641 could target other proteins except for NUCKS upstream of PI3K, and NUCKS1 could modulate the PI3K pathway without miR-641.

## 5. Conclusion

Taken together, these data confirmed that miR-641 exerted tumor-suppressive roles in the development of breast cancer by targeting the NUCKS1-PI3K/AKT pathway.

## Figures and Tables

**Figure 1:** The expression level of miR-641 is decreased in breast cancer cells. The RNA expression level of miR-641 was determined in four breast cancer cell lines (Hs-578T, MCF7, HCC1937, and MDA-MB-231) and a normal breast epithelial MCF-10A cells by real-time PCR and western blotting. ^∗^*P* < 0.05 and ^∗∗^*P* < 0.01, *vs.* MCF-10A cells.

**Figure 2:** miR-641 inhibits the proliferation and promotes apoptosis of breast cancer cells. (a) Detection of transfection efficiency of miR-641 mimics in MDA-MB-231 and MCF7 cells; miR-641 expression was detected by real-time PCR; (b) Green fluorescent in MDA-MB-231 and MCF7 cells under a fluorescence microscope; (c–e) the proliferation abilities of transfected cells were detected by CCK-8 assay, EdU incorporation assay, and colony formation assay; (f) the protein levels of PCNA and Ki67 were measured by western blot; (g) apoptosis detection was performed using flow cytometry; (h) the protein levels of Bax, Bcl-2, caspase-3, and caspase-9 were measured by western blot. ^∗∗^*P* < 0.01*vs.* NC mimics.

**Figure 3:** miR-641 suppressed the migration and invasion of breast cancer cells. (a, b) Migration and invasion capabilities of transfected MDA-MB-231 and MCF7 cells using wound-healing assay and transwell assay; (c) the protein levels of Cox-2, MMP-2, and MMP-9 were measured by western blot. ^∗∗^*P* < 0.01*vs.* NC mimics.

The article "miR-641 Inhibited Cell Proliferation and Induced Apoptosis by Targeting NUCKS1/PI3K/AKT Signaling Pathway in Breast Cancer" was published in 2022. Journal: Comput Math Methods Med.

**Figure 4:** NUCKS1 was a direct target of miR-641 in breast cancer cells. The predicted complementary sequences for miR-641 in the 3′UTR of NUCKS1 and the mutations; (b) miR-641 mimic or inhibitor significantly inhibited or promoted the luciferase activity that carried wt 3′-UTR of NUCKS1 but had no obvious effect on mut 3′-UTR of NUCKS1; (c) NUCKS1 mRNA expression was higher in the bio-miR-641-WT group than that in the bio-NC group after biotin-coupled miRNA sedimentation; (d) NUCKS1 mRNA and protein expression was measured in MDA-MB-231 and MCF7 cells transfected with mimic NC or miR-641 mimics. ^∗^*P* < 0.05 and ^∗∗^*P* < 0.01*vs.* NC mimics or bio-NC.

**Figure 5:** Overexpression of miR-641 inactivates the PI3K/AKT signaling pathway. The western blotting analysis (a) and immunofluorescence (b) were used to detect the levels of the PI3K/AKT pathway in transfected MDA-MB-231 and MCF7 cells. ^∗^*P* < 0.05*vs.* NC mimics.

**Figure 6:** The PI3K/AKT signaling pathway mediates the effect of miR-641 on the breast cancer cells. The cell proliferation (a–c), apoptosis (d), migration (e), invasion (f), and western blot (g) assays in MCF7 cells transfected with miR-641 mimic or mimic NC following treatment with 740Y-P. ^∗∗^*P* < 0.01*vs.* NC mimics and ^##^*P* < 0.01*vs.* miR-641 mimics; ^$^*P* < 0.01*vs.* miR-641 mimics+740Y-P.

**Figure 7:** NUCKS1 overexpression antagonizes the effect of miR-641 on the breast cancer cells. MDA-MB-231 and MCF7 were transfected with either miR-641 mimic or miR-641 mimic in combination with NUCKS1 overexpressing plasmid. (a) Real-time PCR analysis of NUCKS1 in cells transfected with NUCKS1 expressing plasmids. (b) CCK-8 analysis of the cell viability. (c) EdU assay for the cell proliferation. (d) Flow cytometry analysis of cell apoptosis. (e) Transwell chamber assays for the cell migration and invasion. ^∗∗^*P* < 0.01*vs.* NC mimic+vector; ^#^*P* < 0.05 and ^##^*P* < 0.01*vs.* miR-641 mimic vector.

**Figure 8:** NUCKS1 overexpression antagonizes the effect of miR-641 on the PI3K/AKT signaling pathway of breast cancer cells. (a, b) The western blotting analysis was used to detect the protein levels of the PI3K/AKT pathway. ^∗∗^*P* < 0.01*vs.* NC mimic+vector; ^#^*P* < 0.05*vs.* miR-641 mimic vector.

## Data Availability

All data generated or analyzed during this study are included in this published article.
